RETRACTED

# Mosapride Citrate Combined with Divine Qu Disinfectant Oral Liquid for Children Function Dyspepsia and the Influence of Serum Factors

**DOI:** 10.1155/2022/3053277

**Published:** 2022-03-16

**Authors:** Zhenyun Dou, Zhou Xu, Qizheng Wang, Jiangshu Li, Chunlin Yu, Yequan Miao, Tailiang Ren, Haijun Wang

**Affiliations:** ^1^Department of Paediatrics, Huai'an Maternity and Child Health Hospital, Affiliated Hospital of Yangzhou University, Huai'an 223002, Jiangsu, China; ^2^Department of Paediatrics, Hongze District People's Hospital, Huai'an 223002, Jiangsu, China; ^3^Department of Paediatrics, Lianshui County People's Hospital, Affiliated Hospital of Kangda College, Nanjing Medical University, Huai'an 223002, Jiangsu, China

## Abstract

In order to investigate the efficacy of mosapril citrate combined with ShenQu Xiaoshi oral liquid in the treatment of children with functional dyspepsia and the effect on serum cytokines, 136 children with functional dyspepsia admitted from May 2017 to September 2020 were divided into 2 groups randomly, 68 cases in each group. The western medicine group was treated with mosapril citrate tablets, and the combined group was treated with Shenqu xiaoshi oral liquid on the basis of the western medicine group. The efficacy of patients was evaluated 14 days after treatment, and the safety, symptom score, and serum cytokines of the two groups were compared. The results showed that, after 14 days of treatment, the scores of abdominal distension and abdominal pain (ADAP), lack of food (LOF), nausea and vomiting (NAV), irregular stool (IS), and mental fatigue (MF) in the combined group were all lower than those in the western group (*P* < 0.05). There was no statistical significance in the incidence of diarrhea, abnormal liver and kidney, and allergic rash between the two groups (*p* > 0.05). In conclusion, mosapride citrate tablets combined with Shenqu Xiaoshi oral liquid can achieve good therapeutic effects in children with functional dyspepsia, reduce symptom scores, improve serum cytokine levels, and have high drug safety, which is worthy of promotion and application.

## 1. Introduction

Functional dyspepsia occurs in children and refers to persistent or recurrent symptoms such as nausea and vomiting, anorexia, and upper abdominal pain, excluding the syndrome of organic diseases [1, 2]. At present, the clinical pathogenesis of functional dyspepsia in children has not been clarified. It is generally believed that it is related to diet and environment, gastric acid secretion, abnormal digestive tract motor function, etc., which affects children's quality of life and health [3, 4]. Mosapride citrate tablet is a new type of gastrointestinal motility drug, which can act on 5-hydroxytryptamine receptors of neurons and intermuscular nerve plexus, thus effectively promoting gastrointestinal motility and improving gastrointestinal function [5, 6]. According to the symptoms of functional dyspepsia in children, Chinese traditional Medicine dialectics them into the category of “slow lee,” and clinically, according to its etiology and clinical manifestations, it is divided into gastric Yin deficiency, chills and heat, etc. [7]. Shenqu Xiaoshi oral liquid belongs to the common clinical oral medicine of Zhongcheng, which is composed of Shenqu, Hawthorn, and other drugs, and is widely used in diseases such as spleen and stomach weakness. However, there are few studies on the effect of mosapride citrate tablets combined with Shenqu Xiaoshi oral liquid on cytokines of functional dyspepsia in children [8]. In this study, mosapride citrate combined with Shenqu Xiaoshi oral liquid was used to explore the efficacy of functional dyspepsia in children, reported as follows.

RETRACTED

## 2. Materials and Methods

### 2.1. Clinical Data

A prospective analysis was performed on 136 children with functional dyspepsia from May 2017 to September 2020, and they were randomly divided into western medicine group and combined group by random number table method, with 68 cases in each group. In the western medicine group, there were 37 males and 31 females, aged (5–14) years, with an average of 8.95 ± 1.54 years. The course of the disease was 1–4 months, with an average of 2.15 ± 0.53 months. In the combined group, there were 39 males and 29 females, aged from 4 to 15 years, with an average of 8.99 ± 1.61 years. The course of disease was 1–5 months, with an average of 2.19 ± 0.56 months. There was no significant difference in general data between the two groups (*p* > 0.05), indicating comparability. This study was approved by the ethics committee of our hospital and approved by the patients' families. The ethic number is approval no. 2019–55.

### 2.2. Inclusion and Exclusion Criteria

Inclusion criteria:(1) meet the diagnostic criteria of traditional Chinese medicine and western medicine for functional dyspepsia in children [9, 10]; (2) accompanied by persistent or recurrent upper abdominal pain, early satiety, and belching; (3) in line with the indications of mosapride citrate tablet and Shenqu Xiaoshi oral liquid, no history of drug allergy; (4) complete baseline and follow-up data. Exclusion criteria: (1) duodenal ulcer, gastrointestinal bleeding and gastric diseases; (2) congenital malformation, mental disorder, or abnormal coagulation function; (3) antibiotics and other gastric motility drugs were used in the past one month.

RETRACTED

## 3. Methods

After admission, both groups were given routine intervention, instructing the children to eat regularly, defecate regularly, adjust their diet structure, eat more fresh vegetables and fruits, and reduce the intake of meat, carbonated drinks, and snacks as much as possible. Take proper exercise every day and massage your abdomen if necessary. Western medicine group: mosapride citrate tablets for treatment. Mosapride citrate tablet (Chengdu Kanghong Pharmaceutical Group Co., Ltd., National Drug Approval H19990313, specification: 5 mg) 0.2 mg/kg was taken orally, 3 times a day, for 14 days (1 course of treatment). Combined group: based on western medicine group, combined with Shenqu Xiaoshi oral liquid treatment. According to the age of the children, to determine the drug dose, for the age of under 5 years child, each takes Shenqu Xiaoshi oral liquid (Yangtze River Pharmaceutical Group Jiangsu Longfengtang Traditional Chinese Medicine Co., LTD., National drug approval word: Z20153035, specification: 10 mL/bottle) 5 mL, oral, 3 times a day. For children over 5 years old, each takes Shenqu Xiaoshi oral solution 10 mL each time, orally, 3 times a day, continuous treatment for 14 days (1 course).

### 3.1. Observation Index

Symptom score: before and 14 days after treatment, the two groups were evaluated from five aspects: abdominal distension, abdominal pain, insufficient appetite, nausea and vomiting, irregular stool, and mental fatigue, with a total score of 3 points for each item, and the lower the score, the better the effect [11]. (2) Efficiency and security: after 14 days of treatment, patients in the two groups were evaluated in terms of significant effect (all symptoms disappeared, and the score decreased by more than 90.0%), improvement (symptoms improved, and the score decreased by 30.0%–70.0%), and ineffectiveness (the treatment plan was ineffective or needed to adjust the plan) [12]. Response rate = (significant effect + improvement)/total number of cases ^*∗*^100%. The incidence of diarrhea, abnormal liver and kidney, rash, and allergy were recorded. (3) Serum cytokines: interferon-*γ* (IFN-*γ*), tumor necrosis factor-*α* (TNF-*α*), and interleukin-10 (IL-10) were determined by enzyme-linked immunosorbent assay before and 14 days after treatment in both groups.

### 3.2. Statistical Analysis

SPSS24.0 software (SAS, USA) was used for processing, and count data were expressed by *n* (%) *χ*2 test. All the measurement data were in line with normal distribution and were represented by *t*-test. *p* < 0.05 was statistically significant.

## 4. Results

### 4.1. Comparison of Symptom Scores between the Two Groups

There was no statistical significance in the score of symptoms before medication between the two groups (*p* > 0.05). Abdominal distension, abdominal pain, insufficient appetite, nausea and vomiting, irregular stool, and mental fatigue scores in the combined group were lower than those in the western group 14 days after medication (*p* < 0.05), as shown in Table 1.

RETRACTED

### 4.2. The Efficiency and Safety of the Two Groups were Compared

14 d after treatment, the effective rate of combined group was 97.05%, significantly higher than that of western group 75.00% (*p* < 0.05).There was no statistical significance in the incidence of diarrhea, abnormal liver and kidney, and rash allergy between the two groups (*p* > 0.05), as shown in Table 2.

### 4.3. Comparison of Cytokines between the Two Groups

There was no statistical significance of serum cytokines in 2 groups before treatment (*p* > 0.05).The levels of serum cytokines IFN-*γ* and TNF-*α* in the combined group were lower than those in the western group (*p* < 0.05). IL-10 level was higher than that of the western medicine group (*p* < 0.05), as shown in Table 3.

## 5. Discussion

Functional dyspepsia in children is a common disease in children, with clinical manifestations such as abdominal distention and abdominal pain. However, its pathogenesis has not been clarified, and it is generally believed to be related to motor dysfunction, increased gastric acid secretion, and psychopsychological factors [1–14]. Previous studies have shown that [15] children's growing environment can affect the incidence of functional dyspepsia in children. Long-term living and learning pressure, excessive psychological burden, etc., will lead to abnormal gastrointestinal hormone secretion and autonomic nervous dysfunction. In recent years, mosapride citrate tablets combined with Shenqu Xiaoshi oral liquid have been applied in children with functional dyspepsia, and the effect has been satisfactory [16]. In this study, the scores of abdominal distension, abdominal pain, lack of appetite, nausea and vomiting, irregular stool, and mental fatigue in the combined group were lower than those in the Western medicine group at 14 d after treatment (*p* < 0.05), indicating that mosapride citrate tablet combined with Shenqu Xiaoshi oral liquid can reduce the score of functional dyspepsia in children, which is conducive to the recovery of children. Mosapride citrate tablet is a new type of gastrointestinal motility drug with high selectivity. The drug can continuously stimulate the level of enteric intermuscular nerve plexus, thus releasing a large amount of acetylcholine, which can promote gastrointestinal movement, enhance gastrointestinal peristalsis, and improve the gastrointestinal function of children [17].

RETRACTED

In this study, the effective rate of 14 d in the combination group was higher than that in the western medicine group (*p* < 0.05).There was no statistical significance in the incidence of diarrhea, abnormal liver and kidney, and allergic rash between the two groups (*p* > 0.05), indicating that mosapride citrate tablet combined with Shenqu Xiaoshi oral liquid can achieve high efficiency and safety in the treatment of functional dyspepsia in children and can improve the treatment tolerance and compliance of patients. Li Qianwei [18] found that Shenqu Xiaoshi oral liquid combined with mosapride citrate tablets had significant clinical effect in the treatment of functional dyspepsia in children, which was consistent with the results of this study. Liang Yan et al. [19] also came to the conclusion in their study that Shenqu Xiaoshi oral liquid is mainly composed of burnt hawthorn, burnt malt, burnt Shenqu, *Atractylodes atractylodes*, paeony root, amomum, *Poria codonopsis*, Radix xyloderma and Rhizoma corydalis. In recipe, coke hawthorn has blood circulation, disperses stasis, and eliminates product appetizer effect; coke malt has the effect of digestion and hysteresis; Jiao Shen Qu has the effect of invigorating spleen and stomach, digestion, and accumulation; Paeony has the effect of calming the liver and relieving pain, consolidating Yin and preventing perspiration. Tuckahoe can strengthen spleen and prevent diarrhea. *Atractylodes macrocephala* has the function of invigorating the spleen and benefiting the stomach. Dangshen can play tonifying qi and spleen, tonifying lung and shengjin effect; Amomum has the effect of warming spleen and stopping diarrhea, dampening, and appetizing; wood incense can play the effect of adjustment; *Corydalis corydalis* has the effect of invigorating qi and relieving pain. Moxibustion glycyrrhiza can coordinate the effects of different drugs [20]. All drugs, played together, help to improve children's functional dyspepsia symptoms.

The pathogenesis of functional dyspepsia in children is complex and often accompanied by the joint involvement of serum cytokines. Domestic studies have shown [21] that the expressions of IFN-*γ*, TNF-*α* and IL-10 are related to the imbalance of gastrointestinal hormones, resulting in gastrointestinal hypersensitivity and dynamic abnormalities, thus causing functional dyspepsia in children. IFN-*γ* is mainly produced by T lymphocytes and has strong antiviral effect. At the same time, IFN-*γ* can also regulate the immune lymphocyte factor, its expression level can reflect the severity of the disease, TNF-*α* is mainly secreted by macrophages, and its expression level can reflect the body's inflammatory response. IL-10 is a multicell source and multifunctional cytokine that can regulate cell growth and differentiation, directly participates in inflammatory and immune responses, and is recognized as an inflammatory and immunosuppressive factor, playing an important role in infection, hematopoietic system, and cardiovascular system [22]. Serum cytokines IFN-*γ*, TNF-*α*, and IL-10 are in dynamic equilibrium in normal human body, but abnormal expression levels of IFN-*γ*, TNF-*α* and IL-10 will be caused in children with functional dyspepsia. In this study, the levels of serum cytokines IFN-*γ* and TNF-*α* in the combined group were lower than those in western group at 14 days after treatment (*p* < 0.05). The level of IL-10 was higher than that of the western medicine group (*p* < 0.05), suggesting that mosapride citrate combined with Shenqu Xiaoshi oral liquid could improve the serum cytokine level of functional dyspepsia in children. Clinically, mosapride citrate tablet combined with Shenqu Xiaoshi oral liquid can give full play to the advantages of different therapeutic drugs in children with functional dyspepsia, which can help improve serum cytokine level and help control the disease.

RETRACTED

In conclusion, mosapride citrate tablet combined with Shenqu Xiaoshi oral liquid can achieve good therapeutic effect in children with functional dyspepsia, which can reduce the symptom score of children and improve the level of serum cytokines, with high safety and worthy of promotion and application.

## Figures and Tables

**Table 1:** Comparison of symptom scores between the two groups (score).

Group		Abdominal distension abdominal pain	Eat less to stay	Nausea and vomiting	Shit is not adjustable	Mental fatigue
Combined group (*n* = 68)	Before treatment	2.52 ± 0.48	2.51 ± 0.49	2.39 ± 0.42	2.48 ± 0.46	2.44 ± 0.43
	14 d after treatment	0.56 ± 0.15^#^^*∗*^	0.61 ± 0.18^#^^*∗*^	0.73 ± 0.20^#^^*∗*^	0.67 ± 0.16^#^^*∗*^	0.51 ± 0.10^#^^*∗*^

Western medicine group (*n* = 68)	Before treatment	2.54 ± 0.50	2.48 ± 0.46	2.41 ± 0.44	2.50 ± 0.48	2.51 ± 0.49
	14 d after treatment	1.63 ± 0.28^*∗*^	1.68 ± 0.30^*∗*^	1.71 ± 0.32^*∗*^	1.58 ± 0.25^*∗*^	1.61 ± 0.30^*∗*^

Compared with western medicine group, #*p* < 0.05; Compared with before treatment, ^*∗*^*p* < 0.05.

**Table 2:** Comparison of effective rate and safety between the two groups (n (%)).

Group	Number	Efficacy rate			Security		
		Excellent	Improve	Invalid	Diarrhea	Abnormal liver and kidney	Allergic skin rash
Combined group	68	53 (77.94)	13 (19.12)	2 (2.94)	1 (1.47)	0 (0.00)	0 (0.00)
Western medicine group	68	41 (60.29)	10 (14.71)	17 (25.00)	2 (2.94)	1 (1.47)	0 (0.00)
*x* ^2^	—	13.765			1.030		
P	—	0.000			0.310		

RETRACTED

**Table 3:** Comparison of serum cytokines between the two groups (ng/L, $\bar{x}\pm s$).

Group	Number	IFN-*γ*		TNF-*α*		IL-10	
		Before treatment	14 d after treatment	Before treatment	14 d after treatment	Before treatment	14 d after treatment
Combined group	68	2.89 ± 0.54	1.05 ± 0.28^#^	41.56 ± 5.32	21.59 ± 4.19^#^	142.49 ± 14.39	170.67 ± 19.58^#^
Western medicine group	68	2.90 ± 0.55	1.93 ± 0.45^#^	41.55 ± 5.31	32.68 ± 5.03^#^	143.11 ± 14.53	151.49 ± 16.74^#^
T	—	0.107	13.692	0.011	13.969	0.250	6.140
P	—	0.458	0.000	0.496	0.000	0.402	0.000

Compared with before treatment, #*p* < 0.05.

## Data Availability

Data to support the findings of this study are available on reasonable request from the corresponding author.
